# Antimicrobial and anti-biofilm potencies of dermcidin-derived peptide DCD-1L against *Acinetobacter baumannii*: an in vivo wound healing model

This article has been retracted.

**DOI:** 10.1186/s12866-022-02439-8

**Published:** 2022-01-13

**Authors:** Zahra Farshadzadeh, Maryam Pourhajibagher, Behrouz Taheri, Alireza Ekrami, Mohammad Hossein Modarressi, Masoud Azimzadeh, Abbas Bahador

**Affiliations:** 1 Infectious and Tropical Diseases Research Center, Health Research Institute, Ahvaz Jundishapur University of Medical Sciences, Ahvaz, Iran; 2 Department of Microbiology, School of Medicine, Ahvaz Jundishapur University of Medical Sciences, Ahvaz, Iran; 3 Dental Research Center, Dentistry Research Institute, Tehran University of Medical Sciences, Tehran, Iran; 4 Department of Medical Laboratory Sciences, School of Allied Medical Sciences, Ahvaz Jundishapur University of Medical Sciences, Ahvaz, Iran; 5 Department of Medical Genetics, School of Medicine, Tehran University of Medical Sciences, Tehran, Iran; 6 Department of Microbiology, School of Medicine, Hamadan University of Medical Sciences, Hamadan, Iran; 7 Fellowship in Clinical Laboratory Sciences, BioHealth Lab, Tehran, Iran

**Keywords:** *Acinetobacter baumannii*, Antimicrobial peptide, Biofilms, Dermcidin-1L, Wound healing

## Abstract

**Background:**

The global emergence of *Acinetobacter baumannii* resistance to most conventional antibiotics presents a major therapeutic challenge and necessitates the discovery of new antibacterial agents. The purpose of this study was to investigate in vitro and in vivo anti-biofilm potency of dermcidin-1L (DCD-1L) against extensively drug-resistant (XDR)-, pandrug-resistant (PDR)-*,* and ATCC19606-*A. baumannii*.

**Methods:**

After determination of minimum inhibitory concentration (MIC) of DCD-1L, in vitro anti-adhesive and anti-biofilm activities of DCD-1L were evaluated. Cytotoxicity, hemolytic activity, and the effect of DCD-1L treatment on the expression of various biofilm-associated genes were determined. The inhibitory effect of DCD-1L on biofilm formation in the model of catheter-associated infection, as well as, histopathological examination of the burn wound sites of mice treated with DCD-1L were assessed.

**Results:**

The bacterial adhesion and biofilm formation in all *A. baumannii* isolates were inhibited at 2 × , 4 × , and 8 × MIC of DCD-1L, while only 8 × MIC of DCD-1L was able to destroy the pre-formed biofilm in vitro. Also, reduce the expression of genes involved in biofilm formation was observed following DCD-1L treatment. DCD-1L without cytotoxic and hemolytic activities significantly reduced the biofilm formation in the model of catheter-associated infection. In vivo results showed that the count of *A. baumannii* in infected wounds was significantly decreased and the promotion in wound healing by the acceleration of skin re-epithelialization in mice was observed following treatment with 8 × MIC of DCD-1L.

**Conclusions:**

Results of this study demonstrated that DCD-1L can inhibit bacterial attachment and biofilm formation and prevent the onset of infection. Taking these properties together, DCD-1L appears as a promising candidate for antimicrobial and anti-biofilm drug development.

## Introduction

*Acinetobacter baumannii* has become one of the most opportunistic pathogens in clinical settings, especially in patients with infections related to indwelling catheters and burn wound due to the acquisition of resistance genes to most common antibiotics [1].*A. baumannii* as a drug-resistant strain has acquired antibiotic resistance by obtaining plasmids, transposons, or integrons that carry a set of genes encoding multidrug resistance [2]. A prominent ability to accumulate a variety of resistance mechanisms, from inherent resistance to disinfectants to the ability to survive in stressful environments, making this microorganism multi- or pan- drug-resistant, and the ability to develop biofilm, which greatly increases both persistence and resistance in environments, are considered the main features contributing to the survival of this bacteria [3, 4].

The phenomenon of biofilm formation in *A. baumannii* strains is not determined by any single genotype or single factor but is a complex biological and multi-factorial process that is regulated by several bacterial genes. It has been revealed that the expression of several genes to be involved in biofilm formation of *A. baumannii* such as chaperon-usher pilus E (*csu*E), the outer membrane protein A (OmpA), two-component system (*bfm*S/*bfm*R), *Acinetobacter baumannii* autoinducer synthase (*aba*I) and poly-β-(1,6)-N-acetyl glucosamine (*pnag*) [5]. The CsuE is necessary for bacterial adherence and initiation of biofilm formation. Inactivation of the *csuE* gene corresponds to suppression of pilus production and biofilm formation [6]. The bfmRS is a two-component system and regulates the expression of *csu* operon. The bfmRS consists of bfmR as a response regulator encoding gene and bfmS as a histidine sensor kinase gene. The inactivation of bfmS could reduce biofilm formation in *A. baumannii* 17,978 type strain [7]. The OmpA (38-kDa) as an outer membrane protein of *A. baumannii* plays a critical role in bacterial adherence, biofilm formation, and invasion to host cells via interaction with tissue fibronectin. [8]. The AbaI protein (encoded by *abaI* gene) can act as an autoinducer synthase that catalyzes the synthesis of 3-hydroxy-C12-homoserine lactones. Current studies showed that loss of *abaI* gene could result in a significant reduction of biofilm formation and increased antimicrobial susceptibility [9]. Furthermore, the *pgaABCD* locus encodes proteins that synthesize cell-associated poly-beta-(1–6)-N-acetylglucosamine (PNAG). The expression *pga* locus led to the strong biofilm phenotype and antibiotic resistance [10].

Microbial biofilm formation is the critical factor of infection persistence in burn wounds caused by *A. baumannii* [11]. The use of therapeutic approaches such as a combination of debridement by physical or chemical methods, the use of antimicrobial and anti-biofilm compounds, has reduced the incidence of burn wound infections, but there is still the possibility of fatal infections in severe burns, especially in developing countries, which causes an increase the mortality worldwide [12].

Bacteria in biofilm forms are highly resistant to antimicrobial agents compared to planktonic forms [12]. Burn wound infection caused by *A. baumannii* biofilms is the biggest therapeutic challenge, which is treated with polymyxins (i.e. Colistin). However, the mortality rate from *A. baumannii*-associated burn wound infection in patients is very high, especially when the infection is due to multidrug resistant (MDR) *A. baumannii* [13]. Recently, the use of next-generation antibiotics based on natural body-compatible peptides has been developed [14].

Natural antimicrobial peptides (AMPs) as the multi-functional peptides are essential polypeptides in the defense of innate immunity and play an important role in the innate immune system. AMPs as the bioactive small proteins, are divided into two main groups: cationic AMPs and anionic AMPs [15]. They possess broad-spectrum activity against a wide range of microorganisms, including both Gram-positive and Gram-negative bacteria, fungi, parasites and viruses. The unique mechanism of AMPs is related to their cationic and amphipathic properties, which enable them to permeate microbial cell membranes [16].

However, some bacteria have a series of mechanisms to interfere with cationic AMP activity that reduce their attraction to the target site [17]. The active processed form of the human AMP Dermcidin-1L (DCD-1L), as an anionic AMP which is encoded by the DCD gene, could be a potential alternative for evading bacterial resistance against cationic AMPs [18]. Accordingly, one clear advantage of the anionic character of DCD-1L is the ability to circumvent resistance mechanisms that specifically target cationic AMPs [19]. Possibly for that reason, dermcidin is a main effector of the innate host defense against bacterial pathogens, particularly those on human skin [20].

According to the data obtained after a comprehensive literature review, no study exists to evaluate the anti-biofilm activities of DCD-1L. Therefore, in vitro and in vivo assessments of the anti-biofilm activities of DCD-1L against clinical and standard *A. baumannii* strains were performed in this study. In addition, the anti-attachment effect of DCD-1L in the catheter-associated infection model, the wound healing potency in mice with established *A. baumannii* infections, as well as, the effect of this peptide on the expression level of several biofilm-associated genes were evaluated. It was hypothesized that DCD-1L will not only inhibit bacterial attachment and biofilm formation, but also down-regulated the expression level of biofilm-associated genes and improve wound healing.

## Material and methods

### Ethics statement

The present research was approved by the ethics committee of Ahvaz Jundishapur University of Medical Sciences (Ethical code: OG-9742). All experiments in this study were performed in accordance with ARRIVE guidelines (https://arriveguidelines.org).

### Bacterial strains and peptide

One extensively drug-resistant (XDR)-*A. baumannii* and one pandrug-resistant (PDR)-*A. baumannii* with strong biofilm producers which were stored at -80 °C were selected from 100 strains isolated from burn wound infected patients admitted to Shahid Motahari Referral Center of Burn in Tehran, Iran, during 2013–2015 according to our previous study [21]. The XDR-*A. baumannii* strain was resistant to all clinically relevant antibiotics except tigecycline and colistin. PDR-*A. baumannii* strain was non-susceptible to all antimicrobial agents (Table 1).

**Table 1:** The minimum inhibitory concentration (MIC) distribution of 16 antimicrobial agents for the XDR- and PDR-*A. baumannii* strains as determined by E test

*A. baumannii* strains	Antimicrobial agents															
	**PIP**	**TZP**	**SAM**	**CAZ**	**FEP**	**IPM**	**MEM**	**AMK**	**TOB**	**GEN**	**TET**	**MIN**	**TGC**^**a**^	**CIP**	**LVX**	**CST**
**XDR**	≥ 240	≥ 240	32/16	≥ 256	≥ 256	12	24	64	30	30	30	30	0.25	30	10	0.01
**PDR**	≥ 240	≥ 240	≥ 256/128	≥ 256	≥ 256	32	48	256	120	120	30	30	3	60	60	32

*XDR* extensively drug-resistant, *PDR* pandrug-resistant, *AMK* amikacin, *CAZ* ceftazidime, *CIP* ciprofloxacin, *CST* colisitin, *FEP* cefepime, *GEN* gentamicin, *IPM* imipenem, *LVX* levofloxacin, *MEM* meropenem, *MIN* minocycline, *PIP* piperacillin, *SAM* ampicillin/sulbactam, *TET* tetracycline, *TGC* tigecycline, *TOB* tobramycin, *TZP* piperacillin-tazobactam

^a^The minimum inhibitory concentrations (MICs) of *A. baumannii* isolates to 16 antimicrobial agents were carried out using the E test (Ezy MICTM strips, Himedia, India). The Clinical and Laboratory Standards Institute (CLSI) was used for interpretation of the minimum inhibitory concentrations (MICs) results excepted for tigecycline against *A. baumannii* strains. Since there is no breakpoint for tigecycline against *A. baumannii* strains in the CLSI guidelines; therefore, the criteria for interpretation of the MIC values of tigecycline were determined based on the European committee on antimicrobial susceptibility testing (EUCAST; MIC of ≤ 1 mg/L defined as susceptible and > 2 mg/L as resistant)

In addition to clinically isolated strains, *A. baumannii* ATCC 19,606 obtained from Iranian Biological Resource Center, Tehran, Iran was used in our research. The bacterial isolates were inoculated in Luria–Bertani (LB) broth, incubated at 37 °C for 24 h and used for further experimentation. The DCD-1L (purity ≥ 95%) was purchased from proteomics International Laboratories Ltd (PILL), Australia.

### The minimum inhibitory concentration (MIC) and minimum bactericidal concentration (MBC) of DCD-1L

The broth microdilution method was used for determining MIC dose of DCD-1L (Sigma-Aldrich Co., USA) against *A. baumannii* according to Clinical and Laboratory Standards Institute (CLSI) guidelines [22]. Briefly, overnight *A. baumannii* cultures were diluted in fresh LB broth to give a final density of 5 × 10^5^ colony forming unit (CFU)/mL and added to wells of a 96-well polypropylene microtiter plate, containing two-fold DCD-1L-dilutions ranging from 256 to 0.5 μg/mL. The microtiter plate was incubated for 24 h at 37 °C and the MIC was defined as the lowest concentration of peptide at which no growth was observed.

MBC of DCD-1L was determined by re-culturing (subculturing) broth dilutions that inhibit growth of *A. baumannii* (i.e., those at or above the MIC) on Mueller Hinton (MH) agar plates. MBC was defined as lowest concentration of antimicrobial that caused at least 99.999% killing of the initial inoculum [22].

### In vitro evaluation of inhibitory activity of DCD-1L on adhesion and biofilm formation

Inhibitory effect of DCD-1L on biofilm formation of XDR-, PDR-, and ATCC 19,606- *A. baumannii* was analyzed using a static abiotic solid surface assay as previously described [23], with minor adjustment. Briefly, a 200-µL aliquot of 1:100 dilutions prepared from overnight LB culture of *A. baumanni* was added to the wells of 96-well microtiter plates in the presence of different sub-lethal concentrations of DCD-1L (2 × , 4 × , and 8 × MIC) and incubated at 37 °C for 2 h (adhesion assay) and 24 h (biofilm formation assay) without shaking. LB culture of *A. baumanni* without the peptide was considered as a control group. Following incubation, the microtiter plates were washed three times with phosphate buffered saline (PBS) solution and each well was stained with 200 µL of 0.1% crystal violet (CV) for 20 min at ambient temperature. The microtiter plates were again washed three times to remove excess dye. After air drying, CV in each well was solubilized by adding 200 µL of 33% acetic acid (v/v) and the absorbance of the CV was measured at 595 nm (OD_595_) using a microtiter plate reader [23].

### In vitro evaluation of dispersal activity of DCD-1L on biofilms

To perform dispersal activity assay of DCD-1L on existing *A. baumannii* biofilms, initially biofilms were allowed to grow for 24 h at 37 °C in LB medium in a 96-well polypropylene microtiter plate. After biofilm development, DCD-1L at the concentrations of 2 × , 4 × , and 8 × MIC was added to the wells of 96-well microtiter plate and incubated for 12 h at 37 °C. All non-attached bacteria were then removed by discarding the culture medium and rinsing the microtiter plate three times by PBS. Attached biofilm material was stained by 0.1% CV as mentioned above and the absorbance of the CV was then measured at 595 nm using a microtiter plate reader (OD_595_).

### RNA isolation and reverse transcription-PCR (RT-PCR) analysis of biofilm-associated genes transcription

After confirming presence of biofilm-associated genes (*bfmR*, *bfmS*, *csuE*, *ompA*, *bap*, *pgaA,* and *abaI*) by using PCR, the relative expression of these genes in the presence of DCD-1L at 1/2 × MIC was assessed by using RT-PCR. Biofilms were developed in 96-well microtiter plates with and without DCD-1L, as described above. After 24 h of incubation, wells were washed with PBS solution three times to remove planktonic cells and biofilm cells were harvested from the microtiter plates by scraping into RNA protect bacterial reagent (Qiagen, Germany) to stabilize the RNA. The RNA extraction (high pure RNA isolation kit, Roche, Germany) and cDNA synthesis (cDNA synthetic kit, Thermo scientific, USA) were performed according to the manufacturers' instructions. The final concentration of the RNA extracts was adjusted to 0.1 μg/μL. Forward and reverse primer sequences for each gene were designed using Primer Express Software 3.0. These primer sets and their annealing temperatures were listed in Table 2. Quantification of gene transcripts was performed using a SYBR Green PCR Master Mix (Applied Biosystems Waltham, MA) and an ABI Step One Real-Time PCR System (Applied Biosystems) under the following conditions: 95 °C for 5 min, followed by 40 cycles of 95 °C for 10 s, annealing for 10 s at 55 °C, and 72 °C for 15 s [24]. Fold changes in gene expression were calculated using the comparative Ct method (2^−ΔΔCT^) [25, 26] and samples were normalized to *16S rRNA* expression.

**Table 2:** Primer sequences used in this study

**Gene**		**Sequences (5' to 3')**^**a**^	**Product size (bp)**	**Reference**
***ompA***	F	AGCATAAAGAAGCTACACCTGC	154	This study
	R	AAAGTCGCCAAGAAACCTTGAT		
***abaI***	F	CCACACAACCCTATTTACTCGG	121	
	R	GGCGGTTTTGAAAAATCTACGG		
***bfmR***	F	GTGAAGTTCGCCCACACTAT	91	
	R	GCACCCATTTCCAGACCAAG		
***bfmS***	F	GGGCAAAGGCTTCAAATACAC	108	
	R	GGATTACGGGCGGTATTCAT		
***pgaA***	F	TTGATCCAGATGATTAGCGTAGG	99	
	R	AGTCAGGCTAAGGGTGTAGATA		
***pgaB***	F	CGAAGGATATCGCACGTTTC	118	
	R	AATTGGTCAGCACAGGCATT		
***csuE***	F	ACCTTTCTACATACGGCTTCC	104	
	R	CAACTGCGGGTACAGAATAGA		
***16S rRNA***	F	AAAGTTGGTATTCGCAACGG	117	18
	R	ACCTTTAACCCGCTTTTGCT		

*F* forward primer, *R* reverse primer, *bp* base pair

^a^Nucleotides

### Hemolytic activity

In this study, the fresh human blood samples obtained from returned unused blood bags in the blood bank (Iranian Blood Transfusion Organization) were used accordance with the ethics committee. After washing human red blood cells (RBCs) three times with PBS, cells suspension was prepared and incubated for 1 h at 37 °C with serially diluted DCD-1L (at different concentrations: 5, 25, 50, 100, and 200 µg/mL). After centrifugation, the supernatant was collected and the free hemoglobin in the supernatant was analyzed by UV–Vis spectrophotometer at 540 nm. Cells which was incubated with 0.1% Triton X-100 used as 100% hemolysis (control). The hemolysis percentage was calculated as previously described [27].

### Cytotoxicity assay

As described previously [28], 2,3-Bis(2-methoxy-4-nitro-5-sulfophenyl 2H-tetrazolium-5-carbox-anilide (XTT) (cell proliferation kit II, Roche, Germany) was used to determine the cytoxicity of DCD-1L on the mitochondrial activity of human embryonic kidney (HEK)-293 cell line. The HEK-293 cells were grown in DMEM supplemented with 4 mM glutamine, 10% fetal bovine serum (FBS), and 100units/mL penicillin/streptomycin at 37 °C in a 5% CO_2_ and 95% air atmosphere. After 24 h, the incubation medium was discarded and replaced by fresh medium containing various concentrations of DCD-1L (5, 25, 50, 100, and 200 µg/mL). After incubation at 37 °C for 20 min, the medium in each well was replaced by 100 µL XTT reagent mixture and was then incubated for 4 h. Finally, the absorbance was measured at a wavelength of 570 nm using microtiter plate ELISA reader (Anthos 2020, England). The percentage of cell inhibition was calculated using the following formula:

$$\% \mathrm{Cell inhibition} =\frac{\mathrm{Test} \mathrm{Abs }}{\mathrm{Control Abs}}\times 100$$

### In vivo study design and animal care condition

Female Balb/c mice (6–8 week old; 18–22 g) were purchased from Pasture Institute of Iran (Tehran, Iran). All experiments were performed with the criteria described in “Guidelines for Ethical Conduct in the Care and Use of Non-Human Animals” [29]. All mice were housed in single in the small cages, under hygienic conditions at room temperature (22–25 °C) with proper ventilation with convenient access to hygienic water and pellet food. One week before starting the experiments, mice were acclimated to their new conditions. To improve the accuracy of experiments, the cages were disinfected with 10% povidone iodine (PI) solution, and the bedding materials for mice were autoclaved and replaced with new ones every day. In all animal experiments, mice were anaesthetized by intraperitoneal injection of a mixture of xylazine (10 mg/kg) and ketamine (80 mg/kg) and the lower back of each mouse was shaved and cleaned with 10% PI solution.

### In vivo evaluation of inhibitory effect of DCD-1L on biofilm formation in the model of catheter-associated infection

In order to create a subcutaneous pocket to place two 1-cm-long polyurethane catheters, a small incision was made. After implantation of the catheters, injection of a suspension of *A. baumannii* ATCC 19,606 in PBS was performed. The concentration of *A. baumannii* in 250 µL total volume of injection was 10^6^ CFU/mL. DCD-1L were then injected into the subcutaneous pocket of three groups of the animals to get the corresponding concentrations of 2 × , 4 × , and 8 × MIC in total volume of injection (250 µL). In addition, PBS was injected alone to animals as a control group without contamination to evaluate the sterility of surgical procedure. The incision was closed with Vetbond. Tissue adhesive (Kimiatajhiz teb, Iran) and cleansed with 10% PI solution. Mice were sacrificed by an overdose of inhaled isoflurane at days 7 post infection to evaluate bacterial biofilm associated with catheters. Two catheters were removed from each mouse using aseptic technique and catheters-associated biofilms were analyzed by CV assay and scanning electron microscopic (SEM) examination according to the previous study [30, 31].

### Animal model of wound healing

In order to observe the ethics of working with experimental animals based on the Guidelines for Ethical Conduct in the Care and Use of Non-Human Animals in Research [29], after achieving an acceptable test group in the in vitro phase, the in vivo study was done only in that group. Since 8 × MIC dose of DCD-1L showed better anti-biofilm property compared with other groups, this group was selected for animal testing. A 5-mm diameter circular wound was created on the shaved dorsal/ posterior skin of mice as previously described [32]. The mice were divided into two groups and five mice were allocated in each group. The groups were as follows:

a Treated by 8×MIC dose of DCD-1L
b Control (without any treatment)

Five min after generating the wound, DCD-1L was applied on the wound area once daily for ten days. The wound areas were measured on days 0, 1, 5, and 10 using a dial micrometer (Starrett Dial indicator, model 25A, USA), and the contraction rate was determined according to the following formula:

$$\mathrm{\% Rate of contraction} =\frac{\mathrm{Area on day }0-\mathrm{Area on day evaluated }}{\mathrm{Area on day }0 } \times 100$$

### Evaluation of antibacterial effects of DCD-1L on infected burn wound model

The viable bacterial concentrations were determined by colony enumeration of bacterial harvests from the wound area using the biopsy punch method as previously described [32].

### Histopathological examinations of burn wound infections

For histopathological examinations, the mice were treated with DCD-1L at the concentrations of 2 × , 4 × , and 8 × MIC for up to ten days. On the 10^th^ days of treatment, the mice were then sacrificed using 25 and 250 mg/kg of xylazine and ketamine, respectively. As previously reported [32], the wound tissues were removed en bloc and trimmed to include > 0.5 cm beyond the edges. They were immediately fixed in 10% phosphate buffered formalin for 72 h and embedded in paraffin wax. To identify histological changes, 4-μm tissue sections were stained with hematoxylin and eosin (H&E) and analyzed under a light microscope (Olympus, Tokyo, Japan).

### Data analysis

All experiments were performed in triplicate and data are expressed as the mean ± standard deviation. The statistical comparisons between groups were performed using analysis of variance (ANOVA) on the log-transformed data with Tukey–Kramer Honestly Significant Difference Test. The *P* value < 0.05 was considered as significant.

## Results

### Susceptibility of *A. baumannii* isolates against DCD-1L

To determine the antimicrobial activity of DCD-1L against *A. baumannii* isolates the broth microdilution method was used according to the CLSI guideline. According to the results, the MIC and MBC values of DCD-1L against XDR- and ATCC 19,606- *A. baumanni* strains were 16 and 32 µg/mL, respectively, while both MIC and MBC against PDR-*A. baumanni* was 8 µg/mL.

### In vitro anti-adherence and anti-biofilm potencies of DCD-1L

Anti-adherence and anti-biofilm potencies of DCD-1L against *A. baumannii* were determined using colorimetric assay. As presented in Fig. 1a, the bacterial adhesion was significantly inhibited at concentrations which were corresponding to 4 × and 8 × MIC in all *A. baumannii* isolates compared with the control group (*P* < 0.05), whereas the inhibitory effect of DCD-1L at 2 × MIC on bacterial adhesin was only observed for PDR-*A. baumannii* isolate (*P* < 0.05). On the other hand, following treatment with DCD-1L at 2 × , 4 × , and 8 × MIC, significant inhibition in biofilm formation was observed in all isolates in comparison to the control (Fig. 1b; *P* < 0.05).

**Fig. 1:** The inhibitory effects of DCD-1L in different concentrations (at 2 × , 4 × , and 8 × MIC) on a) attachment and b) biofilm formation of XDR-, PDR-, and ATCC 19,606- *A. baumannii* strains using colorimetric assay. *Significant differences according to the control group, *P* < 0.05

### In vitro evaluation of DCD-1L activity in biofilms degradation

The crystal violet biofilm assay was done to detect the biofilms degradation activity of DCD-1L against pre-formed *A. baumannii* biofilms. There was a significant reduction in pre-formed biofilms of all *A. baumannii* isolates (XDR, PDR, and ATCC 19,606) following treatment with 8 × MIC of DCD-1L. As shown in Fig. 2, 128 µg/mL DCD-1L was able to destroy 40.5% and 61.5% of XDR- and ATCC 19,606-*A. baumannii* biofilm, respectively (*P* < 0.05), while a 48% reduction in the PDR-*A. baumannii* biofilm was observed after treatment with 64 µg/mL DCD-1L (*P* < 0.05). DCD-1L at the concentrations of 2 × and 4 × MIC could not destroy biofilm all *A. baumannii* isolates (*P* > 0.05) except concentration 4 × MIC in *A. baumannii* ATCC 19,606 (*P* < 0.05).

**Fig. 2:** The effect of DCD-1L at different concentrations (2 × , 4 × , and 8 × MIC) on biofilms degradation of pre-formed biofilms of XDR-, PDR-, and ATCC 19,606- *A. baumannii* strains using colorimetric assay. *Significant differences according to the control group, *P* < 0.05

Overall, we provide evidence to revealed that biofilms degradation activity of 8 × MIC of DCD-1L against pre-formed biofilm structure of XDR- and PDR-*A. baumannii* as well as ATCC 19,606 strains.

### In vitro biofilm-associated gene expression profiles of *A. baumannii* biofilms

To discover the underlying mechanism of anti-virulence activities of DCD-1L, the gene expression patterns in *A. baumannii* was determined using quantitative real-time PCR. According to the results in Fig. 3, the expression levels of *abaI*, *bfmR*, *bfm*S, *csuE*, and *ompA* genes in isolates treated with 1/2 MIC of DCD-1L were down-redulated by more than two-fold compared to the untreated isolates (*P* < 0.05). Besides, the results indicated that there was no significant reduction in the expression of *pgaA* and *pgaB* genes in the presence of DCD-1L (*P* > 0.05; Fig. 3). Here, we present evidence suggesting that the expression levels of biofilm-associated gene in XDR- and PDR-*A. baumannii* strains were markedly reduced following exposure to DCD-1L.

**Fig. 3:** The expression levels of biofilm formation related genes including chaperon-usher pilus E (*csu*E), the outer membrane protein A (*omp*A), two-component system (*bfm*S/*bfm*R), *A. baumannii* autoinducer synthase (*aba*I) and poly-β-(1,6)-N-acetyl glucosamine A and B (*pna*A/*pna*B) of XDR-, PDR-, and ATCC 19,606- *A. baumannii* strains following exposure to DCD-1L using quantitative real- time PCR. *Significant differences according to the control group, *P* < 0.05

### Cytotoxicity and hemolytic activity assays

To investigate the cytotoxic effect of DCD-1L, the XTT assay was used on HEK-293 cell line. In the current study, hemolytic activity of DCD-1L also was determined using blood cells. The cytotoxicity effect of different concentrations of DCD-1L on HEK-293 cell line was evaluated by XTT assay. According to the results, DCD-1L at the concentrations of 5 to 200 µg/mL had no significant toxic effect on the viability (Fig. 4A) or morphology of HEK-293 cell line compared to the control group (*P* > 0.05; Fig. 4B). In addition, DCD-1L did not exhibit any hemolytic activity against RBCs at the concentrations of 5 to 200 µg/mL (*P* > 0.05). According to present data, DCD-1L was considered a safe and hemocompatible agent.

**Fig. 4:** Cell Cytotoxicity of DCD-1L at the different concentrations on HEK-293 cell line, A) Percent cell viability of HEK-293 cells following exposure to 5, 25, 50, 100, and 200 µg/mL concentrations of DCD-1L using XTT assay. B) A morphometric analysis of cell cytotoxicity using Light-microscopic observations (Mag 40 × , Scale bar 100 µm); a) Control, b) 5 µg/mL, c) 25 µg/mL, d) 50 µg/mL, e) 100 µg/mL, and f) 200 µg/mL

### In vivo inhibitory effect of DCD-1L on biofilm formation in a mouse catheter-associated infection model

We used a mouse catheter-associated infection model, to explore the *in-vivo* anti-biofilm effects of DCD-1L. Based on the data, DCD-1L at the concentrations of 2 × , 4 × , and 8 × MIC significantly reduced the biofilm formation in catheter-associated infection model by 33%, 52%, and 67%, respectively (*P* < 0.05). In order to confirm the biofilm quantification by CV assay, SEM examination was used. Untreated biofilms (Fig. 5a) comprised a denser network of microbial cells and exopolymeric matrix than treated biofilms at 2 × , 4 × , and 8 × MIC of DCD-1L (Fig. 5b-d). Our data revealed that, DCD-1L at the sub-MIC concentrations had an anti-biofilm effect on mouse catheter-associated infection.

**Fig. 5:** Inhibitory effects of DCD-1L at different concentrations (2 × , 4 × , and 8 × MIC) on biofilm formation of *A. baumannii* ATCC 19,606 strain in the mouse model of catheter-associated infection using scanning electron microscopic (SEM) a) Control group, b) 2 × MIC, c) 4 × MIC, and d) 8 × MIC (Scale bar20 microns)

### Efficacy of DCD-1L on wound healing

The contraction rate of wound areas was used to determine the efficacy of DCD-1L on wound healing. The enhancement of wound healing became apparent from a day after the initiation of treatment and most evident after five days. Treatment with 8 × MIC of DCD-1L showed a statistically significant effect on wound closure on days 1, 5, and 10 after treatments in comparison with the control group (*P* < 0.05; Fig. 6). Overall, DCD-1L in a time-dependent manner was promoted wound healing due to contraction rate of wound areas.

**Fig. 6:** Effects of DCD-1L at 8 × MIC concentration on wound healing in infected burn wound model: a) wound closure at different time intervals (0, 1, 5, and 10 days; Scale bar 0.2 cm), and b) Percentage of wound contraction at different time intervals (0, 1, 5, and 10 days)

### In vivo antibacterial effects of DCD-1L on infected burn wound model

To determine in vivo antibacterial effects of DCD-1L on infected burn wound, the viable bacterial counts were determined by colony counting of bacteria harvests from wound biopsies. According to the findings, 8 × MIC of DCD-1L significantly resulted in 1.15, 2.80, and 5.32 log_10_ CFU/mL reductions on days 1, 5, and 10 respectively compared to the control group (*P* < 0.05). The results demonstrated that local effect of DCD-1L at the concentration of 8 × MIC decreased the initial inoculums of *A. baumannii* ATCC 19,606 compared to the control group. Our findings highlight the application of DCD-1L was reduced significantly bacterial counts in burn wound with XDR- and PDR-*A. baumannii* infection.

### Histopathological analysis of infected burn wound

To investigate whether DCD-1L is involved in wound healing process, the evaluation of re-epithelialization, blood vessels, inflammation, and fibroblasts in cross-sectioned tissue obtained from each treated burn wound mice were assessed by the histopathological examinations using HE staining under a general optical microscope. Photomicrographs of normal (a), burned skin (b), and treated burn skin (c-e) stained with H&E are presented in Fig. 7. Complete destruction of superficial skin layers, and Inflammatory changes, signs of coagulation, and infiltration of fibroblasts were observed in burn skin (Fig. 7b). In order to evaluate the wound healing by DCD-1L, histopathological analysis was carried out until the 10th day. As the data show, wound healing with DCD-1L was time dependent. The regeneration in epidermal region with the presence of growing fibroblasts in granulation tissue were shown in the photomicrograph of treated animals (Fig. 7c-e). The proliferation of marginal epithelium was initiated on the 5th day post-treatment (Fig. 7d). On 10th day, continuing re-epithelialization was observed (Fig. 7e). Overall, DCD-1L was markedly involved in wound healing by the acceleration of skin re-epithelialization.

**Fig. 7:** Histopathological sections of the healing incisional wounds following treatment with DCD-1L at different concentrations (2 × , 4 × , and 8 × MIC) for up to ten days using staining by hematoxylin and eosin (H&E; 10 × ; Scale bar 200 µm): a) Normal skin, b) Burn skin, c) Skin tissue treated with 8 × MIC after 1 day, d) Skin tissue treated with 8 × MIC after 5 days, and e) Skin tissue treated with 8 × MIC after 10 days

## Discussion

In this study, biological activity of an anionic AMP (DCD-1L), which as a part of the constitutive innate immune defense of human skin is present naturally in small amounts in the sweat, was examined under in vitro and in vivo conditions. Investigation of antibacterial effect of DCD-1L on opportunistic bacteria revealed strong activity of the peptide against sensitive bacterial strains as well as resistant ones. Schittek et al. demonstrated that antimicrobial activity of DCD-1L occurred in the low μM range. The MIC values reported by them were 1 µg/mL for *Escherichia coli*, *Enterococcus faecalis*, and *Staphylococcus aureus* and 10 µg/mL for *C. albicans*. They indicated that the concentration of this peptide in sweat is 1–10 μg/mL [20]. Interestingly, DCD-1L exhibited an antibacterial effect on the abovementioned pathogens at this concentration range in their study. Likewise, the MIC values of DCD-1L against colistin resistant *A. baumannii* isolates were in this concentration range [21]. Colistin is a cationic lipopeptide and bacteria have acquired resistance mechanism to a cationic lipopeptide by reducing the net negative charge of their surface and reducing, consequently, attraction of the positively charged lipopeptide to the surface; so, this resistance mechanism did not influence susceptibility to the negatively charged molecules such as DCD-1L. These findings are in agreement with the proposed mechanism for DCD-1L by other researchers [33, 34].

Overall, the main antibacterial mechanism of AMPs on planktonic bacteria is the membrane disruption through the electrostatic attraction to negatively charged bacterial surfaces that may result in inhibition of cell wall, nucleic acid or protein biosynthesis [35]. However, the known anti-biofilm mechanism of AMPs is reducing bacterial attachment on biotic and abiotic surfaces, influencing twitching motility, and quorum sensing system [35]. To our knowledge, there are no studies evaluating the anti-biofilm activity of DCD-1L. In the present study, anti-attachment and anti-biofilm activities of this peptide against XDR-, PDR-, and ATCC 19,606-*A. baumannii* isolates showed that the tested peptide was effective against bacterial attachment and biofilm formation of these bacteria. As results showed, 4 × and 8 × MIC of DCD-1L could inhibit bacterial adhesin after 2 h, while 2 × , 4 × , and 8 × MIC considerably prevented the biofilm formation of all isolates after 24 h of incubation. Inhibitory effect on adhesion and biofilm formation was due to its specific inhibitory potency against bacterial colonization. Similarly, AMP-1018 can prevent initial attachment of *Pseudomonas aeruginosa*, *E. coli*, *A. baumannii*, *Klebsiella pneumoniae, Salmonella enterica*, and methicillin-resistant *S. aureus* (MRSA) to surfaces [36].

Several factors cause the bacteria in biofilms up to 1000 times less sensitive to antibiotics than planktonic bacteria. Due to the poor penetration of antimicrobial agents into mature biofilms, the combination of extracellular polymeric substances with antibacterial agents, the efflux effect of efflux pumps, and the presence of persister cells, high-concentration antimicrobial agents should be used to rinse and debride biofilms [37, 38]. In the current study, 8 × MIC of DCD-1L was able to destroy 40.5%, 48%, 61.5% of XDR-, PDR-, and ATCC 19,606-*A. baumannii* biofilm, respectively. Therefore, DCD-1L not only affect initial stages in biofilm formation, but also exerts its anti-biofilm activity by degradation pre-existing biofilm matrix. The important point is that the toxicity and hemolytic activity caused by high-concentration antimicrobial agents must not be ignored. According to the results, DCD-1L at different concentrations up to 200 µg/mL had no significant toxic and hemolytic effects on the viability of HEK-293 cell and RBCs, respectively.

To investigate the underlying mechanism of anti-biofilm activity of DCD-1L, the expression of genes associated with biofilm formation was investigated.

In the presence of the peptide, all biofilm-related genes in *A. baumannii* isolates were significantly down-regulated as compared to control, which may be related to lipopolysaccharide deficiency and weak potency to form biofilm [24], except *pga*A and *pga*B genes. Down-regulation of genes involved in bacterial attachment, *bfm*R and *csu*E, can explain the anti-attachment mechanism to the surface because, the CsuE protein is part of the pili structure in *A. baumannii*, which plays a key role in adhering to the abiotic surfaces and biofilm formation [33]. Binding through *csu*E is the initial and essential stage to produce biofilm on abiotic surfaces. In addition to the *csuE* and *bfmR* genes, the gene encoding OmpA protein was significantly reduced in the presence of DCD-1L, and in addition to pathogenicity, OmpA protein was involved in attaching of this bacterium to biological surfaces (such as the epithelial cell surface) and biofilm formation [33]. Therefore, the anti-biofilm properties of this peptide in the body can also be predicted. Decreased expression level of the *abaI* gene in the presence of this peptide may represent another possible mechanism. The *abaI* gene product is involved in quorum sensing [33], and as we know, quorum sensing is one of the mechanisms involved in biofilm formation [39], and the anti-biofilm properties of DCD-1L can be partially attributed with its anti- quorum sensing property. This is in agreement with previous studies on anti-biofilm effect of LL-37, 1037- AMP, LK6L9 and DJK-5, so that these studies have shown inhibition of biofilm formation by down-regulation of genes-associated in attachment and quorum sensing in drug resistant *P. aeroginosa* [40–43].

As mentioned, it was not observed significant differences in the expression levels of *pga*A and *pga*B genes in DCD-1L treated cells compared to the control. *Pga* locus in *A. baumannii* is associated with synthesize cell-associated poly-β-(1–6)-N-acetylglucosamine (PNAG) which is a major component of biofilms and is essential to maintain biofilm integrity of *A. baumannii* [44].

In the present study, the in vivo anti-biofilm effects of DCD-1L were evaluated on catheter-associated infection. In order to in vivo-evaluation of inhibitory effect of DCD-1L on biofilm formation on catheter, implantation of catheter and bacterial inoculation were performed simultaneously. Our results showed that DCD-1L significantly prevented biofilm development and consequently, reduced total biomass on the catheter at different concentrations of DCD-1L. Since the biofilm development results in protection and survival of bacteria during infection in a hostile environment, the presence of DCD-1L in wound may inhibit biofilm formation and, consequently, help to remove bacteria and promote wound healing.

In vivo investigation of impact of DCD-1L on infected-wound healing showed activity of this peptide in wound closure. Also, the count of *A. baumannii* in infected wounds was significantly decreased following treatment with 8 × MIC of DCD-1L. Histopathological analysis showed that the wound healing with DCD-1L was time dependent. The proliferation of marginal epithelium was initiated on the 5th day and the continuing re-epithelialization was observed on 10th day. In vitro and in vivo infected wound healing activity supported the hypothesis that the peptide not only had a direct effect on bacteria but also had the effects on host through modulating keratinocyte cell migration and proliferation.

The mechanism of wound healing by DCD-1L did not evaluate in this study but previous research demonstrated that DCD-1L does not express on the surface skin of people who suffered from inflammatory skin disorders such as atopic dermatitis, psoriasis, and lichen planus [45, 46]. Dermcidin, unlike to LL-37 as a natural α-defensin was constantly expressed in normal skin and its expression level does not increase in skin inflammation. It seems that DCD-1L with creating conditions for faster wound healing acts as antimicrobial preservative.

## Conclusion

Collectively, our findings showed that DCD-1L affect initial stages in biofilm formation and degradation pre-existing biofilm matrix of *A. baumannii* isolates, as well as, inhibits biofilm formation in catheters without cytotoxicity and hemolytic activity. In addition, DCD-1L deceased the expression of genes involved in biofilm formation of *A. baumannii* and promoted the wound healing by the acceleration of skin re-epithelialization. These effects indicate the preventive role of this peptide on the skin and confirm the protective effect of it in the body, as created by its natural evolution. Collectively, consideration to the available evidence leads us to the conclusion that dermcidin acts as an AMP- rich biofilm layer on skin to prevent bacterial colonization.

## Data Availability

All data was presented in this manuscript.

## Abbreviations

AMP: Antimicrobial peptides
CV: Crystal violet
DCD-1L: Dermcidin-1L
MIC: Minimum inhibitory concentration
MBC: Minimum bactericidal concentration (MBC) of DCD-1L
PI: Povidone iodine
